The article "Slug down-regulation by RNA interference inhibits invasion growth in human esophageal squamous cell carcinoma" was retracted in 2021. Reasons: duplicated images; unreliable results or conclusions; concerns about the images.

# Slug down-regulation by RNA interference inhibits invasion growth in human esophageal squamous cell carcinoma

**DOI:** 10.1186/1471-230X-11-60

**Published:** 2011-05-20

**Authors:** Peng Tang, Zhentao Yu, Kejun Zhang, Yu Wang, Zhongliang Ma, Shaoyan Zhang, Dong Chen, Yanbing Zhou

**Affiliations:** 1 Department of Esophegeal Oncology, Key Laboratory of Cancer Prevention and Therapy, Cancer Institute and Hospital of Tianjin Medical University, Tianjin 300060, R.P. China; 2 Department of surgery, the Affiliated Hospital of medical college, QingDao University, QingDao, Shan Dong Province, 266003. R.P. China; 3 Department of Laboratory, the Affiliated Hospital of medical college, QingDao University, QingDao, Shan Dong Province, 266003. R.P. China

## Abstract

**Background:**

Esophageal squamous cell carcinoma (ESCC) is one of the most aggressive carcinomas of the gastrointestinal tract. We assessed the relevance of Slug in measuring the invasive potential of ESCC cells *in vitro *and *in vivo *in immunodeficient mice.

**Methods:**

We utilized RNA interference to knockdown Slug gene expression, and effects on survival and invasive carcinoma were evaluated using a Boyden chamber transwell assay *in vitro*. We evaluated the effect of Slug siRNA-transfection and Slug cDNA-transfection on E-cadherin and Bcl-2 expression in ESCC cells. A pseudometastatic model of ESCC in immunodeficient mice was used to assess the effects of Slug siRNA transfection on tumor metastasis development.

**Results:**

The EC109 cell line was transfected with Slug-siRNA to knockdown Slug expression. The TE13 cell line was transfected with Slug-cDNA to increase Slug expression. EC109 and TE13 cell lines were tested for the expression of apoptosis-related genes bcl-2 and metastasis-related gene E-cadherin identified previously as Slug targets. Bcl-2 expression was increased and E-cadherin was decreased in Slug siRNA-transfected EC109 cells. Bcl-2 expression was increased and E-cadherin was decreased in Slug cDNA-transfected TE13 cells. Invasion of Slug siRNA-transfected EC109 cells was reduced and apoptosis was increased whereas invasion was greater in Slug cDNA-transfected cells. Animals injected with Slug siRNA-transfected EC109 cells exhihited fewer seeded nodes and demonstrated more apoptosis.

**Conclusions:**

Slug down-regulation promotes cell apoptosis and decreases invasion capability *in vitro *and *in vivo*. Slug inhibition may represent a novel strategy for treatment of metastatic ESCC.

## Background

Despite improvements in detection, surgical resection, and (neo-) adjuvant therapy, the overall survival for esophageal squamous cell carcinoma (ESCC), one of the most aggressive carcinomas of the gastrointestinal tract, remains lower than that of other solid tumors due to distant metastasis [1]. Therefore, efforts are ongoing regarding exploration of novel targets and strategies for the management of ESCC, and gene targeting therapies in particular are promising.

Multiple studies focusing on the effects of various biological factors on the malignant potential of ESCC have been conducted [2-4]. One of those factors is E-cadherin as the loss of E-cadherin is an important step in the process of epithelial-to-mesenchymal transition (EMT) in cancer [5-8].. EMT is an embryonic process necessary for morphogenesis in multi-organ beings. Cells eventually lose E-cadherin and acquire a more mesenchymal, motile phenotype [3,4]. In ESCC, loss of E-cadherin expression is associated with tumor invasiveness, metastasis, and prognosis [2,9-11].

Slug is a member of the snail family of repressors, and is expressed in the neural crest and in mesodermal cells emigrating from the primitive streak in chick embryos [12]. Recently, it has been demonstrated that Slug is involved in the control of apoptosis and in the EMT that is linked to the acquisition of an invasive phenotype [13,14]. Uchikado et al. [11] recently found that E-cadherin and Slug expression were associated with ESCC properties, including depth of invasion, lymph node metastasis, stage, lymphatic invasion, and prognosis. Paras et al. [15] recently reported when the OE33 cell line was is transiently transfected with full length human Slug vector, the expression of E-cadherin was repressed and Slug was negatively correlated with E-cadherin expression. Bcl-2, an apoptosis-related genes, whose expression is Slug dependent in mice [16]. It has been suggested that Slug may be the upregulation gene of bcl-2. Therefore, we believe that blocking Slug expression could be applied to cancer targets.

In this study, we evaluated the effect of Slug blockade and Slug overexpression on survival and invasion in ESCC in vitro and vivo. In a pseudometastatic model of ESCC in mice we demonstrated the existance of an additive effect of Slug silencing in reducing metastatic burden. These data suggest that Slug is a relevant gene for regulation of the metastatic potential of ESCC cells and that Slug inhibition may be suitable as a treatment for metastatic ESCC.

## Methods

### Cell lines

EC109 were kindly provided by Dr. Li (The First Affiliated Hospital, Zhangzhou University, Henan Key Laboratory of Tumor Pathology, Zhangzhou, China). TE13 was obtained from the Japanese Cell Resource Center for Biomedical Research (Sdai, Japan);EC109 cell lines showed the highest level of Slug expression and TE13 cell lines showed less Slug expression [17].

### Slug siRNA construction

Three different double strand siRNA oligonucleotides were successfully made. The sequence was submitted to a Blast search against the human genome sequence to ensure that only the Slug gene was targeted. The following sequences were as followed Sense:5-gatccgcgattgacaccagattcaagagatctgggtactgcattggtcttttttc-3;antisense:5-agctttccaaaaaagaccaatgcagtacccagatctcttgaatctgggtactgcattggtca-3;Sense:5-tgccctcctcacaatagtc tttcaagagaagactattgtgaggagggcttttttc-3;Antisense:5-gatcgaaaaaagccctcctcacaatagtcttctcttgaaagactattgtgaggagggca-3;Sense:5-tgcaaatgtacccaatgatattcaagagatatcattgggtacatttgcttttttc-3;Antisense:5-gatcgaaaaaagcaaatgtacccaatgatatctcttgaatatcattgggtacatttgca-3. A validated medium GC scramble (SCR) double strand siRNA oligonucleotide was used as control for transfection(data not shown). It does not match any mammalian sequences currently available on online databases. The double strand siRNA oligonucleotides were cloned into the pGCL-GFP vector. The pGCL-GFP vectors with double strand siRNA oligonucleotides inserts were used as entry clone vectors and transferred into the vector pDC316-EGFP-U6 [Invitrogen, Carlsbad, CA, USA] using the Gateway *BamH*I and *Hind*III enzyme mix according to the manufacturer's directions [Invitrogen] to generate pEGFP-siRNA-Slug (siRNA-Slug)or pEGFP-siRNA-mock(mock siRNA).

### Slug cDNA construction

The full coding region of human *Slug *(GenBank, AF084243) was amplified by PCR using primers 5'-gctgtaggaaccgccgtgtc-3' and 5'-atttgtcatttggcttcggagtg-3' from cDNA of human EC109 cell line, employing human genomic DNA as the template. The DNA sequence was confirmed and he product was subcloned into the expression vector pGEM-T basic (Clontech, Palo Alto, CA), followed by digestion with BamHI to isolate the BamHI-BamHI fragment of the Slug DNA. The fragment was then subcloned into the vector pDC316-EGFP-U6 [Invitrogen, Carlsbad, CA, USA]and digested with BglII to construct the pSlug cDNA or pEGFP expression plasmid.

### Transcient and stable transfection

The EC109 (TE13) cells were cultured in media for 7 days, plated in a six-well plate with 1 × 10^6 ^cells per well using 2 ml culture medium without antibiotics, and grown to 60-80% confluence for the time of transfection. The Lipofectamine 2000 reagent (Invitrogen; Carlsbad, CA) was used following the protocol set by the manufacturer to transfect the cells with siRNA(cDNA). The following groups were set: [1] RNAi (cDNA) group: the cells were transfected with vector siRNA-Slug(Slug cDNA; [2] Negative transfection group: the cells were transfected with vector siRNA-mock(pEGFP); [3] Control group: the cells were transfected with only liposome and no plasmid. The transfected cells were cultured for 24-72 h, then medium was removed. Stably expressed clones, used for in vivo study and invasion study, were selected by using medium containing G418(250-300 ug/ml) for 28 days. Cells were routinely maintained in selection media containing 200-250 ug/ml of G418-sulfate to avoid overgrowth of nontransfected cells.

### Measurement of Apoptosis

The nucleosomal DNA degradation was quantified by Cell Death Detection ELISA kit using antihistone antibody (Roche, Mannheim, Germany) as described previously [18]. Briefly, 1 × 10^5 ^EC109 or TE13 cells were seeded in 5-cm culture dishes and allowed to adhere overnight. After treatment with siRNA-Slug (Slug cDNA) under the same schedule as described above for 72 h, following which both adherent and floating (apoptotic) populations were harvested. They were lysed in NP-40 lysis buffer and the nucleosomes in the supernatant were detected photometrically using an ELISA plate Reader (SpectraMax 190, Molecular Devices). The readings were expressed as degree of apoptosis considering the untreated control as 1.

To detect DNA fragmentation in cell monolayers after siRNA-Slug (Slug cDNA) treatment, TUNEL was performed by using the *in situ *Cell Death Detection kit (Roche, Inc.) that relies on fluorescent labeling of DNA strand breaks according to the manufacturer's instructions. Positive apoptotic nuclei were recorded by fluorescence microscopy.

### In Vitro Cell Growth Assay

The in vitro growth effects of siRNA-Slug or Slug cDNA on EC109 or TE13 cells were assessed using MTT (Sigma Chemical Co.) Briefly, 1 × 10^4 ^cells were seeded in each well of 96-well microtiter plates and allowed to attach overnight. After treatment with siRNA-Slug (Slug cDNA) under the same schedule as described above for 24-72 h, 20 ml of 5 mg/ml MTT in PBS was added to each well, followed by incubation for 4 hours at 37°C. The formazan crystals were dissolved in DMSO. The optical density was determined with a microculture plate reader (Becton Dickinson Labware, Lincoln Park, NJ) at 540 nm. Absorbance values were normalized to the values obtained for the vehicle treated cells to determine the percentage of surviving cells. Each assay was performed in triplicate.

### Clonogenicity Assay (Soft Agar Assay)

In vitro tumorigenecity and anchorage-independent growth were assayed using standard methods. Stably transfected cells were harvested and suspended in culture medium. One percent agarose was coated onto 35-mm plates, and further overlaid with cell suspension (5,000 cells in 0.5% agarose). Plates were incubated in humidified tissue culture incubator at 37°C, 5% CO_2_, for 2 weeks. Visible colonies were counted under a phase-contrast microscope.

### Quantitative real-time PCR(Q-PCR)

Total RNA was isolated with TRIzol Reagent (Invitrogen) and first strand cDNA was synthesized from 1 ug total RNA using Oligo d(T) primer (Invitrogen) and ReveTra Ace (TOYOBO, Osaka, Japan). Q-PCR was done using 2 ul of first-strand cDNA to quantitatively determine the relative amounts of Slug cDNAs. Primers used were for Slug: F: 5-AGA TGC ATA TTC GGA CCC ACA-3 and R: 5-CCTCAT GTT TGT GCA GGA GAG-3. β-actin, 5-CAA CTG GGA CGA CAT GGA GA-3 and 5-CAG GCA GCT CGT AGC TCT TC-3 [Genebank accession BC_004251]. β-actin was used as internal control in all reactions. Real Time PCR reactions were carried out in triplicate in a volume of 25 μl containing 50 ng of cDNA template,1*× *SYBR Green Mix(Toyobo, Osaka, Japan), and 200 nM or 400 nM of forward and reverse primers. Samples were heated to 95°C for one and a half min, followed by 30 amplification cycles for 30 sec at 95°C and for 30 sec at 65°C for annealing and amplification. Product purity was controlled by melting point analysis. The amount of Slug mRNA was normalized to the endogenous reference β-actin and each experiment of ESCC cell line was used Gene Expression Macro Software (Version 1.1, BioRad).

### Western blotting

Cellular proteins were extracted and separated on SDS-PAGE gels, and Western blotting analyses were carried out as described previously(19). Antibodies used were anti-Slug(G-18:1:200), anti-Bcl-2 (N-19: 1:250) and anti-E-cadherin(G-10: 1:200). All were from Santa Cruz Biotechnology; anti-β-actin (AC-15:1:500) from Sigma-Aldrich.

### Subcutaneous xenografted tumor model

Tumor samples(metastasis node) fixed in 10% neutral buffered formalin were embedded in paraffin using automatic embedding equipment, after which 5-μm sections were prepared. Immunohistochemical analysis for Slug (dilution at 1:100; Santa Cruz Biotechnology)was done on paraffin-embedded sections of mice according to the manufacturer's instruction. After washing with phosphate-buffered saline, the sections were incubated with biotinylated secondary antibody. Positive staining of Slug was seen in the cytoplasm of tumor cells. The results of the immunohistochemical stainings were evaluated by the percentage of positively stained carcinoma cells. TUNEL staining for tumor tissue was based on the protocol of the Dead End Colorimetric TUNEL System (Promega). The tissue sections were viewed at ×100 magnification and images were captured with a digital camera. Percentage of apoptotic cells was defined as TUNEL-positive cells among 1000 tumor cells. Percentage of TUNEL-positive cells in each group were calculated from three tumor

specimens.

### Tumor invasion in Matrigel-coated chambers

The BD BioCoat Matrigel™ invasion chambers with polyethylene terephthalate-filters coated with matrigel basement membrane matrix (6 wells, 8 μm pore size; BD Biosciences, Franklin Lake, NJ) were re-hydrated just before the assay using FBS-free DMEM according to the manufacturer's instructions. The chambers were assembled using freshly prepared matrigel-coated filters and DMEM containing 0.8 mL NIH-3T3 as a chemoattractant in the lower compartment. Stably siRNA Slug transfected or Slug cDNA-transfected cells were harvested by trypsinization, and suspended in DMEM containing 10% FCS. The cells (at a concentration of 1.25 × 10^5 ^cells/2 ml) were added to the invasion chamber containing a matrigel-coated filter. The assembled chambers were incubated for 24 h at 37°C. At the end of the incubation, nonmigrating cells, which remained on the upper surface of the filter, were completely removed by wiping with a cotton swab. The cells on the bottom surface of the filter were fixed with 100% ethanol for 30 sec and stained with toluidine blue for 10 min. Cells migrated in the lower chamber were counted. Experiments were repeated thrice.

### In vivo analysis

Immunodeficient male mice, 4 to 6 weeks old, were purchased from Shang Hai Animal Center. All animals were maintained in a sterile environment and cared for within the laboratory animal regulations of the Ministry of Science and Technology of the People's Republic of China (http://www.most.gov.cn/kytj/kytjzcwj/200411/ t20041108). Autoclaved cages containing food and water were changed once a week. Mouse body weight was measured every 3 to 4 days. On the day of tumor cell inoculation, tumor cells at 60% to 80% confluence were trypsinized and resuspended in fetal bovine serum-free culture medium. Animals were injected in the abdominal cavity with 5 × 10^6 ^cells(siRNA Slug transfected cells, siRNA-mock transfected cells or control cells). The experiments were terminated 21 days. Animals were sacrificed by CO_2 _inhalation, autopsy was carried out for assessment of metastases macroscopically. The number of the seeded tumor in the abdominal cavity is used for assessment of metastases.

### Statistical analysis

All statistical analyses were performed using the SPSS11.0 software. The results were presented as means ± SD of three replicate assays. Differences between different groups were assessed using ANOVA or Dunnett t-test. A *P *value of <0.05 was considered to indicate statistical significance.

## Results

### Slug modulates invasion in ESCC cells in vitro

Recent data indicate that Slug expression is relevant for melanoma metastasis [20]. We undertook experiments to assess whether Slug is involved in ESCC invasion and metastasis. We tested whether Slug knockdown affected the invasion capabilities of ESCC cells by using an *in vitro *invasion assay. In Slug-silenced EC109 cells, invasion was significantly reduced (Figure 1 A). Western blot analysis resulted in Slug protein at significantly lower levels in siRNA Slug-transfected EC109 cells (Figure 1 C, *P *< 0.05). The results indicate that Slug-silence affected the invasion capabilities of ESCC cells. We also tested the effects of Slug cDNA transfection on the invasion capability of ESCC cell line TE13. Expression of Slug was significantly increased in Slug cDNA-transfected cells(Figure 1 D, *P *< 0.05) and the invasion capability was significantly elevated(Figure 1 B, *P *< 0.05). Compared to untreated cells, no further decrease or increase in invasion capability was observed in mock transfected cells. Together, these data show that Slug modulates invasion of ESCC cells *in vitro*.

**Figure 1:** **Slug regulates ESCC cells invasion in vitro**. *A,B, *Stable Slug-transfected EC109 cells or Slug cDNA-transfected TE13 cells(1.25 × 10^5^) were seeded into the upper chamber of the Transwell and the lower chamber was filled with 0.8 mL NIH-3T3 conditioned medium to induce chemotaxis. After 24 h of incubation at 37°C, the cells that invasion through the pores to the lower surface of the filter were counted under a microscope. Three invasion chambers were used per condition. The values obtained were calculated by averaging the total number of cells from three filters.*C,D, *Slug Protein expression was determined by Western blot in stable Slug-transfected EC109 cells or Slug cDNA-transfected TE13 cells.

### Slug affects the in vitro growth of ESCC cell lines by affecting proliferation

This study analyzed the effect of Slug on the cell growth of EC109 and TE13 cell lines. EC109 cell lines were transfected with siRNA Slug, TE13 cell lines were transfected with pSlug cDNA, and their viability was followed for 72 hours using a MTT cell proliferation assay. Cell growth over the 72-hour period for the EC109 and TE13 cell lines transfected with siRNA Slug and Slug cDNA is shown in Figure 2A and 2B, respectively. Each value is measured in triplicate. Significant growth inhibition was found in siRNA Slug-transfected EC109 cell lines compated with mock siRNA control (P < 0.05)(Figure 2A). On the contrary, Slug cDNA promotes growth in TE13 cell lines compated with mock cDNA transfected TE13, although the difference was not significant (*P *= 0.085, Figure 2B). Figure 2A and 2B showed that the growth curves for Slug siRNA-transfected EC109 cells were significantly lower than those for control cells, and the growth curves for Slug cDNA-transfected TE-13 cells were significantly higher than those for control cells. Furthermore, colony formation assay in monolayer culture showed that the number of surviving colonies of Slug siRNA-transfected cells was markedly decreased compared to those of control cells, and the number of surviving colonies of Slug cDNA-transfected cells was increased compared to those of control cells, although the difference was not significant (*P = 0.072*, Figure 2C), suggesting that knockdown of Slug expression inhibits colony formation, and slug overexpression seems to enhance colony formation.

**Figure 2:** **Slug affects proliferation in ESCC cells**. *A,B,*MTT assay was done to investigate proliferation of siRNA-transfected EC109 cells and Slug cDNA-transfected TE13 cells. Every 24 h, the absorbencies of test well were read and semilogarithmic curves were drawn. *Points, *mean of three separate experiments; *bars, *SD. *C,D, *Down regulation of Slug inhibited colony forming ability, and *u*pregulation of Slug promotes colonyforming ability. Histogram was the average number of colonies in each group.

### Slug silencing induces apoptosis in EC109 cells

We evaluated the effects of Slug siRNA transfection on apoptosis induction in EC109 cells using an ELISA kit to quantitatively measure fragmented DNA. After the same treatment schedule described above, a significantly higher level of DNA fragmentation was detected after Slug siRNA transfection compared to those of control cells (Figure 3A, *P *< 0.05). We further evaluated the effects of Slug siRNA transfection on apoptosis induction using an TUNEL kit. After the same treatment schedule described above, a significantly higher level of cell apoptosis index was detected after Slug siRNA transfection compared to those of control cells (Figure 3.B, *P *< 0.05). Western blot shown a significantly higher level of Slug protein in Slug-transfected EC109 cells for 72 h compared with controls (Figure 3 C, *P < 0.05, *P < 0.01).

**Figure 3:** **Effect of Slug silencing on EC109cell apoptosis**. ***A, ***After the same treatment schedule as described above, DNA fragmentation was quantitatively measured by Cell Death Detection ELISA kit using antihistone antibody. Each column represents the mean value of three independent experiments with standard deviation. *Differs from control (P = 0.0043) by Student's t test. ***B***, TUNEL analysis showed a higher percentage of positively stained cells in siRNA-transfected EC109(72 h) compared with control tumors, the difference was significant (*P *= 0.026). Bars, SEM. *, raw values multiplied by 100 for scale. Original magnification, ×200.C, Slug Protein expression was determined by Western blot in Slug-transfected EC109 cells for 72 h(*P < 0.05;**P < 0.01).

### Slug modulates bcl-2 and E-cadherin in ESCC cell line

It has been demonstrated that Slug is involved in the control of apoptosis [14] and also involved in the EMT, linked to the acquisition of the invasive phenotype [19], we analyzed the expression of several Slug targets in stable siRNA Slug-transfected EC109 cells and Slug cDNA-transfected TE13 cells by western blotting and Q-PCR. In siRNA Slug-transfected EC109 cells, anti-apoptotic Bcl-2 was down-regulated (Figure 4 A, *P *< 0.05). By contrast, in Slug cDNA-transfected TE13 cells, Bcl-2 was up-regulated (Figure 4A, *P *< 0.05). E-cadherin, a well-known target of Slug previoussly discribed [20], was up-regulated in siRNA Slug-transfected cells(*P *< 0.05), but in Slug cDNA-transfected cells, E-cadherin was down-regulated (Figure 4 B, *P *< 0.05).

**Figure 4:** **Slug modulates bcl-2 and E-cadherin expression in vitro**. *A, *Q-PCR(top) and western blot (below) analysis for Bcl-2 in stable siRNA Slug-transfected EC109 cells and Slug cDNA-transfected TE13 cells. *B*, Q-PCR(top) and western blot (below) analysis for E-cadherin in Slug cDNA-transfected EC109 and Slug cDNA-transfected TE13 cells.. The experiment was repeated thrice with similar results.

### Effect of Slug silencing in an in vivo pseudometastatic model

We first tested the effect of siRNA Slug-transfected cells in EC109 pseudometastatic models. The mice were injected with stable siRNA Slug-transfected (18 animals) or siRNA mock-transfected (18 animals) EC109 cells(5×10^6 ^)at the site of the abdominal cavity on day 0. After 21 days, the animals were sacrificed and autopsy was carried out to remove organs. Liver metastasis occurred in only four mice in parental groups, and three in mock-transfected mice, no liver metastasis occurred in siRNA Slug-transfected groups. There were many off-white nodus in peritoneum, retina, mesentery, intestinal and gastric wall(Figure 5 A-I, magnification ×200). The node that less than 2 mm is round, and irregular when the node is more than 3 mm. Autopsy showed a reduction of seeded tumor nodes in abdominal cavity organs in pEGFP-siRNA Slug-transfected groups. The number of seeded tumor was 91.16 + 8.7, 90.4 + 9.04 and 33.17 + 6.49 in control groups, siRNA mock groups and Slug siRNA groups respectively. Differences of seeded tumor reached statistical significance (Figure 5 J, *P *= 0.037).

**Figure 5:** **Slug silencing inhibits seeded tumor in a pseudometastatic model of ESCC *in vivo.***. Seeded tumor in abdominal cavity organ(A-F)and Seeded tumor in liver (G-I) of each animal was evaluated for the extent of metastatic invasion. Seeded tumor in abdominal cavity was showed in parental (A)and siRNA mock-transfected mice(B), fewer seeded tumors in abdominal cavity were seen in siRNA Slug transfected mice(C). Seeded tumor in abdominal cavity organ was showed in parental (D)and mock transfected mice(E), fewer seeded tumors in abdominal cavity organ were seen in siRNA Slug transfected mice(F). Seeded tumor in liver was showed in control(G)and mock transfected mice(H), fewer seeded tumors in liver were seen in siRNA Slug transfected mice(I). Significant seeded tumor differences between the control and mock transfected groups are indicated(*P *< 0.05) (J),( magnification ×200).

Furthermore, we analyzed the expression of Slug in the tumor sections from control, mock and Slug siRNA transfected groups using immunohistochemistry (Figure 6 a and 6b). Positive staining of Slug was seen in the cytoplasm of tumor cells. We observed significant Slug expression in control and mock-transfected tumor sections. However, expression levels were drastically reduced in siRNA Slug-transfected sections of mice. TUNEL staining in the same samples was increased from 1.6% positive area in the mock siRNA transfected group to 14.2% positive areas in the siRNA Slug transfected groups(Figure 6 c and 6d).

**Figure 6:** **Immunohistochemical and TUNEL staining in vivo xenograft model**. *A,*Immunohistochemistry with monoclonal antibodies directed against human Slug was performed to compare the Slug expression profile of Slug- and vector-transfected clones in the in vivo human xenograft model. Bars, 21 mm. (a) Slug is intensely expressed in siRNA mock-transfected group.(b)Slug is weakly expressed in siRNA Slug-transfected group, *B*, TUNEL staining in the mock siRNA(c) and the siRNA Slug transfected groups(d).

## Discussion

Esophageal squamous cell carcinoma (ESCC) is one of the most aggressive carcinomas of the gastrointestinal tract, and yet the molecular changes necessary for tumor cells to acquire metastatic competence are still not completely understood.

In addition to the important role during embryonic development, loss of cell adhesion and induction of EMT are required for tumor progression [22]. In fact, induction of EMT represents the first step in the metastatic cascade, allowing cells to delaminate from the primary tumor and to intravasate into lymphatic or blood vessels [3]. Snail, ZEB, and basic helix-loop-helix transcription factors activation represents one molecular switche whereby cells undergoing EMT lose intercellular connections and apico-basal polarity [20]. Recently it has been demonstrated that activation of microRNA-10b by Twist1, an EMT regulator, plays a role in breast cancer invasion and metastasis [23].

Slug is a member of the snail family of repressors, and is expressed in the neural crest and in mesodermal cells emigrating from the primitive streak in chick embryos. Recently, another critical role of Slug has been reported. Slug binds to E-box elements in the proximal E-cadherin promoter and represses transcription of the E-cadherin gene(24). Experimental data have led to the inclusion of Slug into the Snail family of transcription regulators involved in tumor progression and metastasis [11,25]. Previous data suggest that Slug expression significantly correlated with reduced E-cadherin expression in patients with esophageal squamous cell carcinoma, and patients with reduced E-cadherin expression or positive Slug expression have a poor clinical outcome [11].

In our study we found that the knockdown of Slug expression inhibited invasion capability in EA109 cell lines *in vitro*, and overexpression of Slug increased the invasion capability in TE-13 cell lines *in vitro. *It has been reported Slug is involved in cell invasion through direct E-cadherin regulation. We found Slug expression in EC109 and TE-13 cells to show a significant correlation with E-cadherin expression, which is in concordance with the proinvasive role of Slug in EC109 and TE-13 cells.

Zhang et al. [20] has previously found knockdown of Slug expression promotes apoptosis and inhibits cell proliferation in esophageal adenocarcinoma cell in vitro. In the present study, MTT and clonogenicity Assay revealed that overexpression of Slug significantly promotes cell proliferation of the TE-13 cell lines, and Slug inhibition significantly inhibits cell proliferation of the EC109 cell lines. ELISA and TUNEL staining revealed that apoptotic cell death was abundant in EC109 cells with slug inhibition, but almost completely absent in cells transfected with mock siRNA. These data demonstrate Slug silencing gene facilitates apoptosis.

Moreover, Slug is also involved in cell survival through the direct or indirect transcriptional regulation of anti-apoptotic genes [16]. In our studies, we detected a decrease of anti-apoptotic gene Bcl-2 expression in Slug siRNA-transfected EC109 cells, whereas Bcl-2 levels in Slug-cDNA-transfected TE-13 cells increased, findings that demonstrate the anti-apoptotic role of Slug in EC109 and TE13 cells. Although over expression of Slug inhibited apoptosis in TE-13 cells, no statistical significance was demonstrated in control TE-13 cells due to the low apoptosis rate (<5%) (data not shown).

In tumors, migrating cells that leave the primary mass must counteract anoikis [26], a form of apoptotic cell death triggered by the detachment of cells from the extracellular matrix, to arrive successfully at the final site of metastasis. Thus, the anti-apoptotic and proinvasive activities conferred by Slug to ESCC cells *in vitro *could act in concert to promote metastasis competence *in vivo*. To investigate whether the Slug knockdown can synergistically reduce the metastatic burden in ESCC, we used a EC109 pseudometastatic model in immunodeficient mice, Slug silencing did inhibit metastatic growth and the effects reached statistical significance. In the present study, we have investigated the effect of Slug on apoptosis and growth in EC109 cells in vivo. We found that knockdown of Slug expression promotes apoptosis in vivo.

## Conclusions

Our data have shown for the first time the relevant role of Slug expression in apoptosis, invasion and metastasis of ESCC cells *in vitro *and *in vivo*. Although metastasis formation in ESCC as well as in other cancers is a highly complex and organized process that consists of multiple interrelated steps, Slug seems to play a central role, so that its inhibition significantly decreases, albeit does not eradicate, metastasis formation *in vivo*.

## Competing interests

The authors promised there were not any possible conflicts of interest in this research.

## Authors' contributions

TP and YZT participated in the design and coordination of the study and constructed the gene vector; It was TP and YZT to transfect the vector to the cells, carried out the proliferation assay and the apoptosis assay in vitro; ZSY carried out the Q-PCR assay;LXY and WY carried out the in vivo assay. Otherwise, it was TP and YZT to draft the manuscript and performed the statistical analysis. All authors read and approved the final manuscript.

## Pre-publication history

The pre-publication history for this paper can be accessed here:

http://www.biomedcentral.com/1471-230X/11/60/prepub
